The article "Accuracy Assessment of Kriging, artificial neural network, and a hybrid approach integrating spatial and terrain data in estimating and mapping of soil organic carbon" was retracted in 2022. Reasons: compromised peer review; a conflict of interest; concerns about the authorship.

# Accuracy Assessment of Kriging, artificial neural network, and a hybrid approach integrating spatial and terrain data in estimating and mapping of soil organic carbon

**DOI:** 10.1371/journal.pone.0268658

**Published:** 2022-05-26

**Authors:** Miraç Kılıç, Recep Gündoğan, Hikmet Günal, Bilal Cemek

**Affiliations:** 1 Department of Plant and Animal Production, Vocational School of Kahta, Adiyaman University, Adiyaman, Turkey; 2 Faculty of Agriculture, Department of Soil Science and Plant Nutrition, Harran University, Sanliurfa, Turkey; 3 Faculty of Agriculture, Department of Agricultural Structures and Irrigation, Samsun, Turkey; Bahauddin Zakariya University, PAKISTAN

## Abstract

This study aimed to produce a soil organic carbon (SOC) content map with high accuracy and spatial resolution using the most effective factors in the model. The spatial SOC estimation success of Inverse Distance Weighting (IDW), Ordinary Kriging (OK), Empirical Bayesian Kriging (EBK), Multi-Layered Perception Network (MLP) and MLP-OK Hybrid models were compared to obtain the most reliable model in estimating the SOC content. The study area was located in Besni district in the Southeastern Anatolia Region of Turkey. Total of 132 surface (0–30 cm) soil samples were collected from the covers 1330 km^2^ land and analyzed for SOC, lime, clay and sand content and soil reaction included in the estimation models. Mean annual precipitation and temperature, elevation, compound topographic index, enhanced vegetation and normalized difference vegetation index, were also used as the inputs in the modelling. The spatial distribution of SOC was determined using a MLP and a two-stage ensemble model (MLP-OK) combining the estimation of OK residuals. Soil surveys and covariates were used to train and validate the MLP-OK hybrid model. The MLP-OK model provided a more accurate estimation of SOC content with minimal estimation errors (ME: -0.028, 45 MAE: 0.042, RMSE: 0.066) for validation points compared to the other models. The MLP-OK model outperformed other models by 75.09 to 77.92%. The MLP-OK model estimated the lower and upper limits of the estimated and the measured values in a consistent manner compared to the other models. The spatial distribution map of SOC content obtained by ANN-kriging approach was significantly affected by ancillary variables, and revealed more detail than other interpolation methods in the northern, central, southwestern and southeastern parts of the study area. The results revealed that the assembling of MLP with OK model can contribute to obtain more reliable regional, national and global spatial soil information.

## Introduction

The information on spatial distribution of soil properties is important to mitigate the problems on food security, soil quality and land degradation ranging from the local, regional and national to the global level [1–3]. Policies related to the aforementioned problems have been prepared by the utilization of models and possible scenarios, which are an integral part of the spatial soil information [4]. Therefore, the detailed and reliable spatial distribution maps of soil properties are needed for sustainable management of soil resources, and increase the accuracy of environmental modelling outputs. However, most of the available soil maps do not adequately reflect the soil-environment relationship, and composite mapping units of soil maps have insufficient spatial information on soil properties [5]. Therefore, the soil maps produced at high resolution with more details are now of vital importance [6].

The predictive soil mapping and modeling studies are based on commonly accepted soil formation factors. The empirical deterministic soil formation model introduced by Dokuchaev was formulated by Jenny as climate, organism, relief, parent material and time [7,8]. The use of soil formation factors in digital soil mapping has gradually increased with the developments of computer technology [9]. McBratney modified Jenny’s equation and introduced a new soil formation factors equation, also known as SCORPAN [10]. Thus, the accuracy in spatial estimation of soil properties at unsampled points has increased, and more reliable results have been obtained in models explaining the relationship between site-specific soil data and environmental variables. A better understanding of the complex structure of soil ecosystem accelerated the modeling studies [11,12].

Machine learning (ML) techniques using spatial variables and measured values of the attribute of interest are very popular in mapping of soil characteristics. The machine learning algorithms based on various approaches as well as geostatistical methods have been used in soil classification and mapping of soil properties [13–15]. Three different approaches are widely used in mapping soil properties or soil classes. The first approach is statistical machine learning algorithms such as Classification Regression Tree, Support Vector Machines, and Boosted Regression Tree, which stochastically ignore the spatial variation [16–18]. The second approach is geospatial models that model the spatial structure of field observations without considering the deterministic tendency such as kriging [19,20]. The third approach is hybrid models that use spatial variation and statistical models by employing both stochastic and deterministic approaches. The hybrid models have better performance due to their hybrid structure [21]. However, the hybrid models have some disadvantages, for example, kriging and multiple linear regression models in the interpolation and estimation process may result in very high correlation between linearity and mapped soil characteristics and inputs [22]. Therefore, artificial neural network (ANN) technique is used to overcome this problem using limited soil properties and environmental variables [23]. In addition, the main disadvantage of Cubist, Boosted Regression Tree and Random Forest (RF) machine learning algorithms is predicting the values by only considering the decision tree nodes of the auxiliary information at that point, regardless of the spatial autocorrelation of the measured soil properties [24]. Unlike traditional model approaches, the ANN produces powerful results for estimating nonlinear patterns. The ANN compares output and input data during the training process to calculate residual value. The algorithm then returns to the input layer to recalculate weights in the network equation. The success of ANN depends only on the data quality and the architecture of the model. This structure allows to holistically consider the environmental factors affecting the soil property to be predicted [25,26]. Therefore, the paradigm of the current study is to integrate the kriging of the residuals from the ANN into the model, allowing for better spatial estimation while also considering the spatial autocorrelation.

The potential of soils to store organic and inorganic forms of carbon has a greater impact on climate change and global warming than atmospheric carbon [17]. The management of soil organic carbon (SOC) is very important both due to the active role in reducing the atmospheric greenhouse gases concentration on a global scale, and the positive effects on improving soil quality on a local scale. [27]. Therefore, SOC is one of the most widely used indicators of soil security and soil quality assessment [28]. Sustainable management of SOC is a key mechanism for improving soil functionality and delivery of soil related ecosystem services [29]. Therefore, the main motivation of the presented study is to obtain the most accurate estimation of SOC content, and prepare a spatial distribution map by improving the current methods used in digital soil mapping.

The SOC is a spatially highly variable soil property, while easy to measure. Therefore, estimation of SOC content in areas larger than a single field might be quite difficult. The spatial variation of SOC content is closely related to pedogenic factors, vegetation and topography [30]. Climate, primarily the effects of temperature and precipitation, have a significant impact on the SOC content and mineralization rate. The temperature is an important factor controlling the decomposition rate of plant residues. For example, every 8–9°C increase in annual mean air temperature almost doubles the mineralization rate [31]. In addition, the SOC content increases with the increase in the annual average precipitation [32]. Most of the changes in SOC content in a landscape are related to changes in plant species and density. For example, herbaceous vegetation produces a large root mass compared to the above-ground component, while most of the organic matter in forests is produced on soil surface, and the residues are more resistant to the decomposition [33]. The altitude which is a topographic variable, is more likely related to variation in texture and mineralogy of soils due to the changes in geology, and the temperature of the location [34]. Therefore, the selection of the parameters to be used in a model to determine the temporal and spatial distribution of the SOC content is very important. In addition, the relationship between the variables affecting the SOC storage is not linear but hierarchical [35]. Therefore, the ability to accurately determine the SOC spatial distribution in large areas is closely related to the relationship between the soil forming factors and the input parameters in the study area.

The objectives of the study are (i) to produce a high spatial resolution SOC map to develop effective policies on problems of land degradation, and soil and food security at a local scale; (ii) to include the most effective and the least number of factors to the model, considering the hierarchical structure of the factors affecting the SOC, without compromising the estimation accuracy; (iii) to compare the spatial SOC estimation success of Inverse Distance Weighting, Ordinary Kriging (OK), Empirical Bayesian Kriging, Multi-Layered Feed-Forward Backpropagation Network (MLP) and MLP-OK Hybrid models; and (iv) to develop a mathematical MLP model to practically estimate the SOC content under similar conditions of the study area.

## Material and methods

### Study area

This study was carried out in Besni district of Adıyaman province in the Southeastern Anatolia Region of Turkey (Fig 1). The study area is located between 37° 41’ 34 " North latitude and 37° 51’ 40" East longitude, and covers 1330 km^2^ land. Long-term (2001–2021) annual average temperature of the study area is 17.7°C and the average precipitation is 636 mm [36]. The study area consists of Mesozoic aged limestone, marl and schist units. In addition, locally various ophiolitic groups and alluviums are located on the valley floors and around the streams. The geomorphological structure in the study area is essentially a karstic plateau fragmented by small rivers. The elevation decreases from west to east, and there are many poljes and uvalas in the plateau of the study area. The important rivers are Göksu River, Aksu River, Sofraz Stream and Karasu Streams, which all merges to the Euphrates River [37].

**Fig 1:** Geographical location of the study area and spatial distribution of the train and test dataset used for the model.

The study area’s soil temperature regime is mesic, while the moisture regime is xeric. The soils in the study area are belonged to the Inceptisols, Vertisols and Entisols orders according to Soil Taxonomy [38]. There is no problems of drainage, salinity and alkalinity, and only light to moderate stoniness on the surface and in the profile and shallow soil depth on sloppy areas [39].

Natural vegetation: It consists of plants such as wild pistachio, hawthorn, wild pear, bitter almond, turmeric, sandalwood tree, mulberry. Also, there are degraded oak forests as well as maquis in Besni. Grapes, peanuts, wheat, barley, lentils, and chickpeas are widely grown in the polje, uvala plains and mountainous hilly areas in the western part of the study area. Almond and olive cultivation have also increased recently on the valley floors and wide plains irrigated from various streams. Likewise, various vegetables and fruits such as walnuts, apricots, mulberries, and cherries are also grown in irrigated areas.

### Soil sampling and environmental variables

The study area was divided into 4 x 4 km square grids for soil sampling. The soil samples were collected in 2021 from approximately the corners of each grid. In addition, 11 fine transects with 100, 500, 750 and 1250 m intervals were sampled to determine the spatial variability within shorter distances than 4 km, and to increase the success of the model presented in the study. Total of 132 surface (0–30 cm) soil samples were collected from the study area. The location, latitude and longitude of each sampling point were recorded in the field using a global positioning system (GPS). The soil samples were dried, ground, passed through a 2 mm sieve and prepared ready for laboratory analysis. The texture of the soil samples was determined by the hydrometer method [40]. The lime content was determined using the Scheibler calcimeter’s carbon dioxide output volume [41]. Soil pH was measured in a 1/2.5 (soil/water) mixture using a pH meter [42]. Organic matter content of samples was analyzed using the Walkley–Black dichromate oxidation procedure [43].

Digital elevation map of the study area was prepared using the 12.5 m resolution ALOS-DEM downloaded from the Alaska Satellite Facility Distributed Active Archive Center [44]. The datasets are freely available to the public at the ALOS PALSAR RTC Initiative official website (https://search.asf.alaska.edu/#/) [45]. The elevation from west to east of the study area changes between 1200 and 1500 m, and this part of the study area has the characteristic of a sloping plateau. The lowest elevation (400 m) is the valley floor where the Göksu Stream emerges to the Euphrates River in the southeast, and the highest location (1510 m) is the Akdag hill in the northwest [46].

Compound Topographic Index (CTI) transformation, alternatively referred to as the "soil wetness" transformation, can be used to simulate various aspects of hydrologic systems. The CTI is directly proportional to soil moisture, and is a characteristic of both the slope and the area upstream of the flow direction per unit width orthogonal to the flow direction. The CTI was developed specifically for hillslope catena [47], and calculated as follows [48];

$$CTI=\frac{Ln\alpha }{Lnß}$$ (1)

Where; α denotes the area of the catchment per unit width orthogonal to the direction of the flow, and ß denotes the slope.

The data for annual average precipitation and temperature were downloaded from the Meteorological Data Information Presentation System of General Directorate of Meteorology [36]. The precipitation data of the last 20 years from 26 meteorological stations and around the study area were mapped using the IDW kriging method [49]. The temporal variation of the climate data indicated that most of the precipitation occurs in the winter and the study area has a precipitation regime similar to the Mediterranean climate. The precipitation starts in October and increasingly continues until April. The least rainfall occurs in July and August, and the highest precipitations occur in December, February, and March. The precipitation is sufficient in spring and winter seasons for plant growth, while insufficient in summer seasons; therefore, the lack of precipitation in summer months leads to drought and increases the need for irrigation in agriculture.

### Spectral indices

The Sentinel-2A images for December 2020 and June 2021 were downloaded from the European Space Agency (ESA) as remote sensing data to retrieve the spectral indices. The image is freely available at Sentinel Scientific Data Hub (https://scihub.copernicus.eu). The median of Sentinel-2A satellite images for bare soil periods (December 2020) and green periods of cultivated areas (June 2021) were used to decrease the weak observation effect and obtain more accurate soil surface reflection [50].

The spectral index is an efficient and quick means of generating model input variables [51]. Enhanced vegetation index (EVI) and normalized difference vegetation index (NDVI) were used as vegetation indexes in the study [52,53]. The NDVI and EVI are plant indices that allow spatial estimation of soil organic matter and organic carbon and characterize vegetation information [54,55]. The vegetation indices can reduce the spectrum errors, and thus improve the accuracy of SOC estimation [56]. The equations used to calculate the EVI [50,57] and NDVI [50,58] are as follows (Eqs 2 and 3)

$$EVI=2.5x\frac{b_{8}-b_{4}}{b_{8}+6Xb_{4}-7.52b_{2}+1}$$ (2)

$$NDVI=\frac{b_{8}-b_{4}}{b_{8}+b_{4}}$$ (3)

In the equations; EVI is the enhanced vegetation index, NDVI is the normalized difference vegetation index. b8, b4 and b2 are the NIR, red and blue bands of Sentinel 2, respectively.

### Spatial prediction of SOC content using multi-layered feed-forward backpropagation network

The maps of soil properties and environmental variables used as the input data in the SOC estimation model were created as a GIS database within ArcGIS. All layers from different sources were organized in the same projection system.

The sampling points were randomly divided into two groups using the “create subset” function in Geostatistical Analyst of ArcGIS 10.8 (Fig 1). Seventy percent (n = 90) of the sampling points was used for training the ANN model and 30% (n = 42) was for validation of the outputs (Fig 1). The minimal dataset used to report the results have been given in S1 Table.

A multilayer feedforward backpropagation artificial neural network (MLP) with input variables was used to increase the estimation accuracy of SOC mapping. The MLP is a back propagation machine learning consists of an input layer, one or more hidden layers, and an output layer. The first layer of MLP is the input layer, which consists of input variables of the model. The last layer is the output layer, which consists of the output results, and the layers between the input and output layers are known as hidden layers. Following the description of the general structure of the MLP, the model needs to be trained. Levenberg-Marquardt backpropagation training algorithm was used for training in the study. Levenberg-Marquardt is a network training function that updates the weight and bias values according to the optimization. This algorithm is highly recommended, although it requires more memory than other algorithms [59–61].

The structure of the final ANN model used to predict SOC is shown in Fig 2 Soil properties (clay, sand, pH and lime), remote sensing data (NDVI, EVI), mean annual precipitation and temperature, elevation and CTI were used as the inputs of the ANN model. Each of the ANN model input is connected to a hidden layer with a tangent sigmoid transfer function (Eq 4) with their optimal weights. The resulting output was the SOC value predicted by the ’purelin’ linear transfer function.

**Fig 2:** The structure of the ANN model used in the study. ’tansig’ tangent sigmoid function; ’purelin’ represents the linear transfer function.

The ANN has 10 inputs and 14 hidden layer neurons. The weights of the inputs (*X1*, *X2*,*…*..*X10*) and the connections between the inputs and the hidden layer were presented in the *W* matrix. The elements of the *W* matrix are *wi*,*j; i = 1*,*2*,*…*,*10;and j = 1*,*2*,*…*.,*14*, which is the weight between the input unit i. and the neurons j. The *bh*_*1*_, *bh*_*2*_ ……., *bh*_*14*_ are the bias values for 1., 2.,……,14. hidden layer neurons, respectively. The vector *V* represents the weights between the hidden layer units and the output layer. The *b*_*01*_ is the side value for the output layer [62].

In artificial neural networks, it is possible to model nonlinear relationships using activation functions. The hyperbolic tangent activation function (tansig) is one of the most frequently used activation functions in artificial neural networks. To use this function, the input values must first be normalized to the range (-1,1), and the output values must also be normalized to the range (-1,1) [63]. Tansig is remarkably advantageous, which is presented for application, because we want the outputs to be between (-1,1) following the normalization process [64]. The tansig transfer function was calculated using the following equation [63];

$$tansig(x)=\frac{2}{1+\exp\left(-2x\right)}-1$$ (4)

In the equation; x is the ’tansig’ transfer function and is defined where x represents the corresponding input.

The parameters such as the number of hidden neurons in the network system were determined during the trial and error process. The data used in the training process of the model had different units; therefore, they were treated equally to improve the performance of the training network. The data were normalized in the range of 0–1 to reduce the dimension [65]. The development process of MLP-ANN model was carried out using MATLAB R2021a software. The data obtained from field and laboratory studies and remote sensing data of the sampling locations were used in the MLP training. Then, the equation obtained from MLP was transferred to the GIS environment using the "raster calculator" tool in ArcGIS 10.8 software and mapping was performed.

### Estimation of residuals with ordinary kriging

The ANN estimation was carried out in the residual kriging procedure. The residual error of a point was calculated using the following equation (Eq 5);

$$r(x_{i})=Z(x_{i})-{Ẑ}_{ANN}(x_{i}),$$ (5)

In the equation; *r(xi)* is the residue at *xi; Z(xi)* is the actual value at point *xi*, and *Ẑ*_*ANN*_*(xi)* is the value estimated by the MLP. The spatial structure was preserved in the new *r(xi)* variable, while the effect of complex environmental variables was eliminated by the difference between *Z(xi)* and *Ẑ*_*ANN*_*(xi)*.

In addition, the spatial trend in Ẑ_*ANN*_(xi) values was disappeared by the effect of MLP. The data used in the study had a spatial trend, therefore, successful predictions were obtained by applying another geostatistical estimator (kriging) to the residuals after such trend removal procedure. Similar procedure has been applied by Dai et al. [66], Demyanov et al. [67], Seo et al. [68] and Song et al. [69].

The *r(x*_*1*_*)*, *r(x*_*2*_*)……*,*r(x*_*N*_*)* residues at *x*_*1*_, *x*_*2*_, *……*,*x*_*N*_ points were estimated by ordinary kriging (Eq 6). The ordinary kriging is the most common type of spatial estimation method and the error variance is minimized by ordinary kriging [70].


$${ř}_{OK}{(x}_{0})=\sum_{i=1}^{n}\lambda r(x_{i})$$ (6)

In the equation; *řOK* is the estimated residual value of the ANN at point *xi* with ordinary kriging. The ordinary kriging is equal to *∑λi* under optimal conditions.

The spatial distribution and trend of the data are determined using the experimental semivariograms that measure the mean difference between the data, separated by a lag distance h. The semivariogram is calculated as half the mean square difference between data pairs (Eq 7) [71].


$$Ῠ(h)=\frac{1}{2N(h)}\sum_{i=1}^{N(h)}{\left[r(x_{i})-r(x_{i}+h)\right]}^{2}$$ (7)

In the equation; N(h) is the number of sampling pairs separated by a delay distance h. The model was also used for kriging interpolation of MLP residues [71]. ArcGIS 10.8 software was employed to estimate the residuals in the study area using ordinary kriging.

The SOC content, Ẑ(*xi*), was estimated using the ANN estimates Ẑ_*ANN*_(*xi*) and the sum of the ordinary kriging estimates of the residues [66].


$$Ẑ(x_{i})={Ẑ}_{ANN}(x_{i})+{ř}_{OK}(x_{i})$$ (8)

The predictive maps were created with other interpolation methods (Empirical Bayesian kriging and IDW) and then their prediction accuracies were compared to verify the MLP-Ordinary kriging hybrid approach presented.

### Accuracy assessment using MLP-ordinary kriging hybrid interpolation method

The validation of model was carried in two stages; initially the accuracy of the MLP-OK model was assessed, and later the success of the presented hybrid approach was assessed by comparing the outputs with other interpolation methods.

#### Performance (error) criteria of the MLP model

Root Mean Square Error (RMSE) was introduced to compare the final predicted output with the target output, and a network performance indicator was calculated from the differences between the network output and the target. High RMSE value indicates a lower accuracy in the prediction. The RMSE value, which is inversely proportional to the prediction accuracy was calculated as follows [72];

$$RMSE=\sqrt{\frac{1}{n}\sum_{t=1}^{n}{\left(E_{i}-M_{i}\right)}^{2}}$$ (9)

In the equation, the RMSE is the mean square root of error, E*i* and M*i* are the estimated and measured values, and *n* is the number of samples.

The MAPE (Mean Absolute Percent Error) introduced apart from this criterion [73];

$$MAPE=\frac{1}{n}\sum_{t=1}^{n}|\frac{M_{i}-E_{i}}{M_{i}}|X100$$ (10)

In the equation, *n* is the number of samples, M*i* and E*i* are the measured and estimated values, respectively.

#### Criteria for hybrid interpolation method error

The mean error (ME), mean absolute error (MAE) and root mean square error (RMSE) defined by Isaaks and Mohan [74] to evaluate the performance of different interpolation methods were calculated using the Eqs 11–13.


$$ME=\frac{1}{n}\sum_{i=1}^{n}\left[Ẑ{(x}_{i})-Z(x_{i})\right]$$ (11)

$$MAE=\frac{1}{n}\sum_{i=1}^{n}\left|Ẑ(x_{i})-Z(x_{i})\right|$$ (12)

$$RMSE=\sqrt{\frac{1}{n}\sum_{t=1}^{n}{\left[({Ẑ(x}_{i})-{Z(x}_{i})\right]}^{2}}$$ (13)

In the equations; the *Ẑ(xi)* is the estimated SOC content, *Z(xi)* is the measured SOC content, and *n* is the number of samples used for validation.

Comparison of the MLP-Ordinary Kriging hybrid approach with other interpolation methods for sample points using measured real values was carried out with the relative improvement (RI) (Eq 14) [75].


$$RI=\frac{{RMSE}_{int}-{RMSE}_{MLP-OK}}{{RMSE}_{int}}X100\%$$ (14)

In the equation; RMSE_*MLP-OK*_ and RMSE_*int*_ are the root mean square errors of the multi-layered feed-forward backpropagation artificial neural network and ordinary kriging hybrid approach, and a specific interpolation method used in the study, respectively.

## Results and discussion

### Descriptive statistics of input data used in the modeling

Descriptive statistics of the soil properties, climate characteristics and vegetation indices at the sample points used in the modeling are given in Table 1. The skewness of soil organic carbon (SOC) content at the training and test points was 1.10 and 1.01%, respectively. Positive skewness is an indicator of considerably high SOC values, which are an integral part of the data set, thus were included in the model. The SOC content in the training and test datasets ranged from 0.66 to 2.86% and from 0.50 to 3.42%, respectively. The sampling points with high SOC content in the training and test datasets were located in the highest annual average precipitation of the study area. Likewise, Feng et al. (2002) [76] stated that the effect of precipitation on SOC stocks and content was significantly higher compared to average temperature, altitude and evapotranspiration. In addition, the sampling points with a higher SOC content than the mean SOC value had a higher clay and lime content than the mean clay and lime content. Therefore, high clay and lime content of the soils in the study area con be considered as a positive indicator of SOC stocks. The soil organic matter mineralizes more rapidly in noncalcareous soils than in calcareous soils. Heavy soil texture slows the mineralization of organic matter. In contrast, areas with sandy soil texture had a low SOC content. High surface area of clay soils provide more surfaces to bind SOC, and aggregation preserves organic matter from decomposition [77].

Land use type of sampling points with high SOC content was mainly oak, while conventional wheat production with intensive soil tillage using moldboard plough has been used for a long time at low SOC sampling points. Organic carbon losses under long-term conventional tillage systems have been reported in Mediterranean region of Turkey [78,79]. In addition, low SOC stocks were located mostly in the intensively tilled high clayey soils. Similarly, Bruun et al. [80], reported that total SOC content in Vertisols dominated by smectite type clay minerals after 20 years of intensive cultivation decreased by 40% compared to the no-till natural vegetation land use type.

The distribution of SOC data was slightly skewed, therefore, the median value (1.32 and 1.34%) of the training and testing areas better represented the mean SOC pool compared to the arithmetic mean of the study area [75]. The sampling points included all land use types as well as all the continues variables (precipitation, temperature, elevation, CTI, NDVI, EVI) of the study area (Table 1).

**Table 1:** Descriptive statistics of soil properties, climate characteristics and vegetation indices at sampling points.

Test Data (n = 40)											
	SOC (%)	Clay (%)	Sand (%)	pH	Lime (%)	Temp. (°C)	Prec. (mm)	CTI	Elevat. (m)	NDVI	EVI
**Mean**	1.44	46.82	23.80	7.81	20.17	17.54	52.02	7.91	732.73	0.44	0.31
**Median**	1.34	47.73	23.01	7.81	16.71	17.36	52.73	6.93	727.00	0.40	0.28
**Std. Deviation**	0.56	9.64	9.88	0.17	15.89	1.40	3.04	2.77	171.58	0.18	0.14
**Skewness**	1.10	0.15	0.89	-0.32	0.72	4.00	-0.23	1.36	0.11	0.30	0.56
**Kurtosis**	2.40	-1.05	0.58	0.06	-0.46	21.38	0.22	1.19	-1.10	-0.87	-0.68
**Min**	0.50	30.59	6.51	7.36	1.84	16.20	46.16	4.82	469.00	0.11	0.09
**Max**	3.42	66.01	50.85	8.10	59.80	25.06	58.54	15.45	1078.00	0.79	0.61
**Coefficient of variation**	39.08	20.59	41.52	2.12	78.75	7.96	5.84	35.01	23.42	41.45	44.35
Train Data (n = 92)											
**Mean**	1.36	45.34	26.68	7.74	19.37	17.54	52.11	7.83	703.02	0.50	0.35
**Median**	1.32	44.67	24.73	7.72	12.11	17.70	52.41	6.75	707.50	0.48	0.31
**Std. Deviation**	0.42	9.22	11.24	0.19	16.36	0.64	2.36	2.91	129.91	0.16	0.14
**Skewness**	1.01	0.16	0.38	-0.10	0.66	-0.38	-0.14	1.65	-0.03	0.29	0.63
**Kurtosis**	1.57	-0.87	-0.13	-0.30	-0.95	-0.96	1.15	2.03	-1.05	-0.90	-0.47
**Min**	0.66	27.43	4.72	7.29	2.45	16.20	46.16	4.78	438.00	0.21	0.13
**Max**	2.86	65.15	55.50	8.13	58.72	18.54	58.54	17.86	937.00	0.82	0.67
**Coefficient of variation**	31.10	20.33	42.10	2.50	84.49	3.66	4.52	37.20	18.48	32.53	38.96

### Architecture of the MLP network

The relationship between soil and environment variables in digital soil mapping can be explained by using linear models with a few standard soil properties and environmental factors. However, the relationship between three or more factors and soil property and environmental variables can only be explained using advanced models such as non-linear machine learning algorithms, ANNs or fuzzy logic due to the non-linear and unstable relationship between soil properties and environmental variables [81–84]. An MLP network was developed to both increase the accuracy of estimation and reveal the relationship between SOC content and environmental factors by using many environmental variables as well as soil properties (Fig 1). The network was trained using 70% of the observation data, and the success of the network was tested using 30% of the data. The developed MLP network can be explained by the following equation (Eq 15):

$$Predicted\;SOC\;Content=\sum_{k=1}^{K}(([\frac{2}{1+exp(-2(\sum_{i=1}^{K}\sum_{j=1}^{L}\left(\omega_{i}(i,j)X\;{input}_{i}(j))+v_{j}(i)\right)}-1])X\;b_{h}(j))+b_{O_{1}}$$ (15)

In the model equation; *ω* is the weights of connections between inputs and hidden layer, *v* is the weights between hidden layer unit and output layer, *b*_*h*_ is the bias value for hidden layer neurons (Table 2), and *b*_*O1*_ is the bias value for output layer (2.196). The developed MLP model will be practical to predict the SOC content by determining only the input data in different regions with similar characteristics.

**Table 2:** Weight and bias values between the input layer and the hidden layer, and the hidden layer and the output layer.

Number of neuron	IW										Bias	*V*_(1,14)_
	Clay	Sand	pH	Lime	Temperature	Precipiation	CTI	Elevation	NDVI	EVI		
**1**	0.241	0.018	19.404	0.631	-5.517	-2.154	2.774	0.063	10.218	15.217	-5.272	-0.571
**2**	-0.525	-0.080	-3.420	0.316	1.403	-0.312	0.394	0.034	6.428	-13.034	-1.490	-0.870
**3**	0.320	0.495	14.413	0.000	0.407	-1.902	0.074	-0.036	2.338	9.466	-21.002	1.113
**4**	1.764	1.785	-1.559	-0.417	-3.141	3.580	2.265	-0.301	-5.116	0.310	21.625	-0.688
**5**	-0.805	-1.579	-0.054	-0.362	0.189	0.792	0.900	0.092	1.927	1.708	3.019	0.790
**6**	-0.014	0.020	0.846	-0.011	-0.535	-0.033	-0.036	0.000	3.990	-0.286	6.619	-0.181
**7**	0.283	0.190	1.095	0.070	0.905	0.051	-0.373	0.004	-13.875	9.429	-47.684	-0.810
**8**	0.227	-0.298	-2.627	0.188	0.713	-0.342	0.694	-0.001	-2.363	-1.460	10.606	0.933
**9**	1.997	-0.404	0.771	1.000	-2.505	1.807	1.091	-0.283	0.888	-3.802	-10.257	0.882
**10**	0.025	-0.053	-0.530	0.060	0.316	-0.197	0.072	0.022	8.687	-2.382	-14.403	1.171
**11**	-0.024	0.087	-1.613	-0.104	-0.520	0.206	-0.333	-0.007	-12.940	12.850	24.875	1.573
**12**	-0.404	-1.143	-6.161	-0.671	2.706	2.087	-2.373	-0.139	-2.558	20.348	23.717	-0.635
**13**	0.625	-0.169	1.259	-0.811	1.431	0.057	0.505	-0.067	-3.563	-2.057	-2.916	-1.212
**14**	-1.626	0.282	-0.157	0.808	-0.920	0.687	1.350	-0.019	-2.595	-1.484	-5.859	1.167

### Performance of the MLP network

The MLP network was established in MATLAB, and the network was trained using the soil properties and environmental variables of the training points. The test data set was used to determine the optimum selection of activation function, number of hidden layers and other parameters of the model. The final structure of the model was determined during the calibration stage, when the MSE (0.012) and RMSE (0.109) values were the most appropriate according to the information obtained from the literature and trial and error method. The graph of the measured and estimated values of the MLP is given in Fig 3 [23,65,85].

**Fig 3:** Measurement, estimated values, and residual values.

The Mean Absolute Error (MAE) may not always clearly indicate the relative size of the error. Therefore, distinguishing a major error from a minor error may be sometimes difficult. The MAE was calculated as a percentage to deal with this problem [86]. If the MAPE value is less than 10%, the model is considered to have high accuracy (highly accurate forecasting), if the value is between 10 and 20%, the model is moderately accurate (good forecasting), and if the value is between 20 and 50%, the is considered to have low accuracy (reasonable forecasting). If the value is above 50%, the model is considered to have inaccurate forecasting [73]. The Mean Absolute Percent Error (MAPE) value in the model was 4.210%, which indicated high accuracy in SOC estimation.

### Spatial estimation of soil organic carbon content

After the MLP network has been constructed for the study area, the final SOC content was calculated as the sum of the estimated values of the network, and the residual values estimated by ordinary kriging [87]. The residual values for the training points were determined using the Eq 5. The Kolmogorov-Smirnov (K-S) test indicated that the train dataset had normal distribution (p>0.05). However, the distribution of ANN residuals was not normal, thus a square transformation was used [88]. The residuals were used to calculate the semivariogram for the ordinary kriging interpolation following the transformation. The weights of the semivariogram parameters were estimated by the least squares method [89]. The parameters of the most suitable model are shown in Table 3.

**Table 3:** Semivariogram model parameters for soil organic carbon (SOC) content and residual ordinary kriging interpolation in training areas.

Variogram	Model	Range (m)	Nugget	Sill	Nugget/Sill (%)	Root Mean Square
**SOC**	Gaussian	5965	0.121	0.137	88.3	0.277
**Residual SOC**	J-Bessel	1438	0.166	0.775	21.4	0.046

The nugget/sill ratio was used to identify spatial dependency classes of SOC content [90]. The nugget/sill ratio ≤ 25% indicates that the variable is strongly spatially dependent; If the ratio is between 25 and 75%, the spatial dependence is moderate, and if the ratio is >75%, the spatial dependence is weak. The nugget/sill ratio of residual values at training points indicated a strong spatial dependence (21.4%). The spatial dependence was weak (88.3%) in the measured SOC values, while the spatial dependence increased in the residual SOC values (Table 3). The results showed that residual values maintain their spatial characteristics. In addition, this can be accepted as an indicator of the success for the presented methodology when the effect of very complex environmental factors affecting SOC content is eliminated with the ANN and only spatial effect is in question [68,69,87].

Likewise, Abdulwaili et al. [91] reported the spatial dependence of soil organic matter for surface soils in the Manas basin as 68% and Budak and Gunal [92] as 49.7% in upper Tigris Basin in Turkey when interpolated using the exponential model. The results support that soil chemical and biological properties such as SOC have moderate or weak spatial dependence due to their highly dynamic nature.

Predicted SOC content maps obtained by the interpolation methods used in this study revealed the spatial variation of SOC content in the study area (Fig 4). In particular, the SOC content map produced by the MLP-OK hybrid method was significantly affected by the use of auxiliary variables. The high variability of SOC in the study area can be attributed to the differences in precipitation and altitude, as well as agricultural practices such as tillage, crop production pattern, fertilization and irrigation among the sampling points [92]. The comparison of interpolation methods revealed that combination of MLP OK provides a more precise estimation and explains more details than using only ordinary kriging, IDW and Empirical Bayesian Kriging methods especially in the middle of the study area, in the V-shaped zone with high SOC content. Compared to the SOC map produced with the MLP-OK hybrid method, the map closest to the lower value of the SOC content was obtained by the IDW method, while the map closest to the upper value was obtained by the Empirical Bayesian Kriging method. However, both the IDW and the Empirical Bayesian Kriging methods employed only the information on spatial variation of SOC content when producing the spatial distribution maps. Four different soil characteristics, spectral indices reflecting vegetation characteristics, altitude, compound topographic index, temperature and precipitation were considered in the MLP-OK hybrid method, therefore, the lowest and highest value ranges were very close to the actual values determined by laboratory analysis. All models indicated very low SOC content in the south-eastern part of the study area where mainly irrigated agriculture and intensive tillage have been carried out for a long time, which has also been confirmed by the field observations. Organic matter addition to the soils is insufficient in this section, and the mineralization rate is high due to intensive tillage and the prevailing climate, therefore, organic matter decomposed, and the SOC content was lower than other areas [93,94].

**Fig 4:** Soil organic carbon (SOC) content maps obtained using different interpolation methods (4a, 4b, 4c, and 4d are the predicted SOC maps for MLP-OK, OK, IDW, and EBK, respectively.).

The samples were divided into 4 elevation groups (400–650 m, 650–800 m, 800–950 m, 950–1100 m) to reveal the relationship between the SOC content and the elevation of the sampling points. The difference in SOC content between elevation groups is shown in Fig 5. The line on the quadrant groups, where the altitude difference in each box area was separated, shows the median values. The analysis of variance, used to reveal the difference between SOC means in elevation groups, showed that the difference in SOC content was significant (p<0.05) between at least two means. The mean SOC content (1.21%) in the lowest elevation group was significantly (p<0.05) lower than the mean SOC content (1.58%) in the highest elevation group (Fig 5). Similarly, [34] stated that different elevation levels explain most of the variability in SOC content.

**Fig 5:** Soil organic carbon (SOC) content in different elevations.

### Accuracy assessment for the interpolation methods

The indices used to assess the accuracy of the estimated SOC content by all estimation methods and in all test points are given in Table 4. The ME, which expresses the mean bias of the predictions, shows the difference in estimated value from the actual values for all the methods. The underestimation occurred in the ordinary kriging (-0.077) was significantly decreased in MLP-OK (-0.028) method. The ME values show that the low estimates compared to the actual mean SOC content were recorded in IDW (-0.091) and Empirical Bayesian Kriging (-0.067) methods. The MAE, which expresses the absolute value of the difference between the estimate and the actual value, expresses the size of error produced by the model compared to the actual value. The mean difference between the SOC content estimated by MLP-OK method and the actual SOC values was 0.042, which was the lowest value among the prediction methods. The RMSE, a common measure of bias in the mean and variance [95], was greater than MAE values in all methods. This indicates a significant effect of error on spatial variability of the attribute investigated [96,97]. The MLP-OK hybrid method compared to the other methods produced less errors in estimating SOC content with a much lower RMSE (0.042). The RI, indicative of the relative improvement in the RMSE, ranged between 75 and 78%. The results showed that the accuracy of ANN interpolation (RMSE 0.109) was slightly improved with the residual kriging.

**Table 4:** Accuracy assessment of indices (error metrics) at validation points for SOC content estimated using different interpolation methods.

Methods	Accuracy Indices			
	ME	MAE	RMSE	RI (%)
**MLP-Ordinary Kriging**	-0.028	0.042	0.066	
**Ordinary Kriging**	-0.077	0.402	0.277	76.17
**IDW**	-0.091	0.417	0.299	77.92
**Empirical Bayesian Kriging**	-0.067	0.392	0.265	75.09

The Taylor diagram is used to show the quality of model predictions against observed (reference) values (Fig 6). The diagram is used to assess the degree of agreement between estimated and measured data using three different statistical parameters. The statistical parameters used in the diagram are Pearson correlation coefficient (r), RMSE and standard deviation cumulative frequency diagram. Thus, the accuracy of the model simulating the natural system can be visually demonstrated [65,98]. The reference point shown red in the Taylor diagram represents the observed SOC points where the correlation is 1 and the centered root mean square error (CRMSE) is 0. The red line represents the standard deviation of the reference point. The OK, IDW and EBK are located in the left of the red line. The result indicated that the simulated SOC has lower variation, while the MLP-OK above the line shows similar variation with the observed data. The other useful information from the Taylor diagram is the correlation between the SOC interpolation models predicted values and observation values. The MLP-OK hybrid method is located between 0.95 and 0.99 sectors and has a higher correlation than other models. The OK is in the sector of 0.2 and has the lowest correlation. The EBK and IDW are located in the same sector (0.4). The CMRS, which gives an information on the reliability of the modeling process by attaining higher weights to the outliers, was expressed with black, red, green and blue contours. The MLP-OK is in the 0.2 black contour, which shows that the MLP-OK hybrid method has the most reliable modeling process. The OK, IDW, and EBK are pretty close to the green (CMRS 0.6) contour, which indicates that a large number of outliers are generated during the interpolation process [99].

**Fig 6:** Demonstration of performances of different SOC interpolation models with Taylor diagram.

The methodology significantly improved the accuracy of spatial distribution mapping for SOC content. Other interpolation methods, which could not adequately reflect local variations, either overestimate low values or underestimate high values. This problem was significantly corrected both by using the nonlinear model and by taking the factors influencing the SOC content into account. In addition, the results showed that the spatial distribution of soil properties can be successfully estimated with machine learning algorithms by using remote sensing data and environmental variables. The finding confirmed that, similar to the conclusions of Zhang et al. [100], ANNs can be used to interpret the nonlinear relationship between SOC content and ancillary variables. In addition, the spatial distribution map of SOC content generated by ANN-kriging was significantly affected by the auxiliary variables and revealed more details than other interpolation methods in the northern, central, southwestern and southeastern parts of the study area. Previous studies also reported that the ANN successfully reveals local variation in the spatial distribution of SOC content [66]. In summary, the ANN-Kriging hybrid approach compared to conventional interpolation methods is a digital soil mapping model that enables to obtain high resolution SOC mapping, showing local variations, by successfully estimating the SOC content.

## Conclusions

In this study, the accuracy of Inverse Distance Weighting (IDW), Ordinary Kriging (OK), Empirical Bayesian Kriging (EBK), Multi-Layered Feed-Forward Backpropagation Network (MLP) and MLP-OK hybrid estimation models were tested to determine the spatial distribution of soil organic carbon content (SOC) in Besni district of Adiyaman province, Turkey. The accuracy of residual MLP-OK hybrid model to estimate the spatial distribution of SOC content at the regional scale was higher than the other estimation methods tested. The interpolation methods were compared with the MLP-OK model to evaluate the prediction accuracy. An optimal MLP architecture was prepared with three hidden layers, tansig activation function and purelin output function in accordance with the selected pedological and environmental factors for the SOC content estimation. Spatial dependence of MLP residuals was strong. The SOC content map produced with MLP-OK revealed more details than OK, IDW and EBK, especially in the south-central part of the study area, where intensive agricultural practices are carried out.

The Taylor Diagram showed that the MLP-OK model had a lower RMSE and a higher Pearson correlation coefficient for the test sampling dataset. The RMSE value improved between 75 and 78% compared to other methods. The results indicated that estimating the MLP residuals with OK improves the spatial estimation accuracy. In addition, the lower and upper limits of the estimated and measured values were more compatible in the SOC map produced by MLP compared to the interpolation models that only consider the spatial variability. Because the MLP uses many factors such as soil properties, topography, and biota in the estimation process. The MLP-OK method reduced the spatial prediction errors at the local scale SOC content mapping, which requires more attention compared to the other soil properties. The result confirms that the MLP-OK hybrid method can be used as an effective method in digital soil mapping and may contribute to digital soil mapping efforts at regional, national, and global scales. In addition, the study showed that data quality and model architecture are of great importance for the ANN to produce successful prediction models. The findings indicate that in SOC model studies, it is possible to reduce the size of input data without negatively affecting model success. In this context, the use of input such as humidity coefficient, drought coefficient and climate coefficient, which represent many environmental factors, may increase the estimation ability of the models.

## Supporting information

S1 Table Minimal dataset of the study used to analyze, report, and interpret the results. (XLSX)
